The article "Relationship between perceived occupational stress and psychological well-being among secondary school heads in Khyber Pakhtunkhwa, Pakistan" was retracted in 2025. Reasons: duplicated data; duplicated text; overlap with earlier publications; unreliable data.

# Relationship between perceived occupational stress and psychological well-being among secondary school heads in Khyber Pakhtunkhwa, Pakistan

**DOI:** 10.1371/journal.pone.0208143

**Published:** 2018-12-12

**Authors:** Qaiser Suleman, Ishtiaq Hussain, Saqib Shehzad, Makhdoom Ali Syed, Sadaf Ayub Raja

**Affiliations:** 1 Institute of Education & Research, Kohat University of Science & Technology, Kohat, Khyber Pakhtunkhwa, Pakistan; 2 Department of Education, Abdul Wali Khan University, Mardan, Khyber Pakhtunkhwa, Pakistan; 3 Department of Education, University of Kotli, Azad Jammu Kashmir, Pakistan; 4 Department of Education, University of Haripur, Haripur, Khyber Pakhtunkhwa, Pakistan; Universitat de Valencia, SPAIN

## Abstract

The purpose of the study was to examine the relationship between perceived occupational stress and psychological well-being among secondary school heads in Khyber Pakhtunkhwa. A sample of 402 secondary school heads (male *n* = 260, female *n* = 142) was selected through multistage sampling technique. A descriptive, quantitative and correlative research design was used. For gathering information from the participants, two standardized tools i.e., “Occupational Stress Index (OSI)” and “Ryff’s Psychological Wellbeing Scale (RPWB)” were used for measuring perceived occupational stress and psychological well-being respectively. For statistical analysis, mean, standard deviation, Pearson’s product-moment correlation and multiple regression were employed. The findings revealed that there is a strong negative correlation between perceived occupational stress and psychological well-being. Furthermore, moderate negative correlation was found between all the sub-scales of perceived occupational stress and psychological well-being. All the subscales of occupational stress except low status were found significant predictors and have negative effect on psychological well-being of secondary school heads. So, it was suggested that Elementary & Secondary Education Department Khyber Pakhtunkhwa should have a collaboration with policy makers to formulate a comprehensive strategy for stress reduction management for secondary school heads so that they may develop good psychological well-being and perform their duties effectively.

## Introduction

Effective leadership has long been considered very imperative to ensure successful performance of schools by introducing a vivacious environment, providing adequate resources, and creating good relations and students’ performance [1–2]. Social changes have converted the school into a more dynamic and complex institution than what has been experienced so far. A good leader mobilizes resources to achieve the objectives of the collective interests; takes decisions to achieve societal goals; extracts, produces and distributes channels towards the promotion of indiviudal’s prosperity in the organization. Due to the importance of leadership in the community, heads may provide effective leadership for the attainment of educational goals. It is imperative to modify and improve the perfomrance of the school head and to recognize specific leadership behaviors and practices that have positive effects on instiutional as well as as students’ performance [3].

The article "Relationship between perceived occupational stress and psychological well-being among secondary school heads in Khyber Pakhtunkhwa, Pakistan" was retracted in 2025. Reasons: duplicated data; duplicated text; overlap with earlier publications; unreliable data.

Successful leaders are aware of their feelings and knows the strengths and weaknesses, and they have a strong sense of self-respect and self-esteem. Effective leadership manage themselves with discipline, control negative emotions, show flexibilities, and maintain integrity. A head of the school must use emotional as well as general intelligence to accomplish these responsibilities to meet effectively the mandates of state and federal as well as fulfil the mission and the vision of the school successfully [2]. Therefore, effective leadership is widely accepted as being a fundamental element of an organization and playing a vital role in ensuring individuals’ prosperity and organizational productivity. Without effective leadership, an organization cannot succeed in getting right way of success and leaders are unable to perform their duties effectively until they are psychologically strong, competent, satisfied and secured in a working place. Leaders having problems may create numerous disagreeable and unpleasent consequences for organization and its workforces which pessimistically affect the overall performance of an organization. Therefore, psyhcolgoical well-being and occupational stress of individuals are the most dominant and leading variables as these variables are directly responsible for good and bad performance.

### Occupational stress

Occupational stress has gained more attention in the recent years, as the number of employees experience it increasingly since globalization takes place. An occupationally upsetting environment drives an organization toward devastation and obliteration. An occupationally stressful leader fails to ensure fulfilling the productive and gainful outcomes in an organization. Occupational stress takes place due to professional variables relating with the employees to adjust their psychological and physiological conditions which usually cause the mind or body of the individual to go amiss from its normal functioning. Research has revealed that turnover rates of the working forces increase when occupational stress increases. Therefore, occupational stress contributes to a number of difficulties and hindrances to organization in the shape of non-attendance, loss of efficiency and poor health resources. The notions i.e., occupational stress, organisational stress, job stress, and work-related stress are conceptualized interchangeably on the grounds that occupation, job, work and organisation are commonly indistinguishable concepts. Occupational stress is a kind of emotional, behavioural and physiological reactions to foreboding and disparaging aspects of working environment, work association and working conditions. The main accentuation is given on the work environment as it goes about as the wellspring of stress [4]. Occupational stress is unending condition caused by the conditions in workplace that tangles antagonistically influences on the workers’ employment progress and their general thriving. Occupational stress is interminable condition created by the conditions in workplace that can belligerently influence the employment progress of the employees and their general prosperity [5]. Occupational stress alludes to the disagreeable physiological and psychological consequences that rise in individuals because of their powerlessness to oversee and satisfy the demands being forced on them. It is caused by the mutual connection of individuals, or as a result of managing organizational plans and environmental conditions [6].

The article "Relationship between perceived occupational stress and psychological well-being among secondary school heads in Khyber Pakhtunkhwa, Pakistan" was retracted in 2025. Reasons: duplicated data; duplicated text; overlap with earlier publications; unreliable data.

There are numerous factors that contribute to occupational stress in working situation. A number of research studies have explored different underlying causes contributing to occupational stress in various organization such as, workload, conflicts among workers and organizations, role ambiguity, undesirable and disappointing interpersonal relationships, customer contact, job independence, locus of control and social support. Different factors that are leading and powerful stressors composed of five events yielding stress i.e., home-developed issues and demands, family-based issues, marital issues and clashes between family demands and employment [7]. The stressors which are constantly perceived in the literature are workload, time pressure, educational change, investigation, leadership styles, innovation, re-organization, and insufficient resources. Investigating the causes of occupational stress, Willis [8] documented stressors as anxiety, narcissism, hate, guilt feelings, over-sensitivity, desire, sufferings, frustration, terror, disappointment and yearning for endorsement. In addition, he laid out methods of change events which add to extreme stress i.e., personal injury or aliment, demise of life partner, divorce, wedding, sex issues, pregnancy, gain of a new family member, issues with supervisors, issues with managers, monetary commitments, change in working conditions, changes in school and minor infringement of the law. Among these, sexual harassment and belligerent behavior at home are the important sources of stress. The underlying causes for stress in workplace comprise of maltreatment, feeling weak and uninvolved in choosing one’s own responsibilities, harassment, lack of viable communication, lack of effective conflict resolution, unreasonable performance demands, instability of employer, politics among staffing, long working hours, passing more time away from family, a feeling that one's compensation is not equivalent with one’s responsibilities, and pressures disturbing life-balance [9]. Occupational stress may be caused due to extraordinary or too little work, time pressure, deadlines and physical strain created by the working place and its conditions. Employment environment likewise goes about as hotspot for making social and psychological stress [10].

The article "Relationship between perceived occupational stress and psychological well-being among secondary school heads in Khyber Pakhtunkhwa, Pakistan" was retracted in 2025. Reasons: duplicated data; duplicated text; overlap with earlier publications; unreliable data.

Occupational stress is a noteworthy issue with organizational management and leadership. Stress contributes to problems like unsatisfactory performance, family issues, poor social relationships, health problems and unproductive organization. Although the outcomes of stress are different relying upon the circumstances and attributes of the people involved, the outcomes for the people are reliably unexpected. Depression, anxiety, downheartedness, tension and disappointment are conceivable results. Stress has unfavorable effects on the prosperity of the employees. Occupational stress is a global and frequently has recognized a debilitating human phenomenon. Stress that takes place in the working environment has harmful effects on employees’ behaviour which ultimately effect personal and organizational productivity negatively [10]. Among numerous occupational antagonistic impacts of work stress are employment dissatisfaction, poor social relationships, decreased profitability, non-attendance; high staff turnover; nervousness, depression, and burnout [11]. Perceived occupational stress is reported to have adverse and pessimistic effect on mental health, as measured by insomnia, depression, psychological well-being, anxiety, happiness, etc. [12]. Consistent extraordinary level of occupational stress can bring about veritable wellbeing conditions including hypertension, cancer and mental diseases, for example, downheartedness or downfall. Stress has adverse effects on the organization as well as individuals’ mental and physical condition which bring about unsatisfactory performance, non-attendance, accidents, dishonest conduct, discontentment and sickness [13]. In a nutshell, occupational stress can be classified into three classes i.e., psychological strain, physical strain and behavioural strain.

The article "Relationship between perceived occupational stress and psychological well-being among secondary school heads in Khyber Pakhtunkhwa, Pakistan" was retracted in 2025. Reasons: duplicated data; duplicated text; overlap with earlier publications; unreliable data.

Psychological strain is the main type of strain which is caused by stressors which also known as psychological health. Strain refers to the abnormality from normal reactions and psychosocial strain includes reactions i.e., job dissatisfaction, anxiety, melancholy, low self-regard and unsettled issues [14]. A huge assemblage of literature proposes that work stress is firmly identified with nervousness and downheartedness. Encountering of stress is associated with the mental areas of exhaustion, depression, low self-respect, outrage, lethargy, touchiness, blame, ill-temperedness, accidents, fatigue, withdrawal and burnout [15–16]. Psychological strain comprises of dissatisfaction, apprehension, tension, dysphoria, sleeping disorder, impatience and restlessness [17]. The outcomes of stress might be of emotional appearances–feelings of indistinct nervousness, disappointment, discouragement, fear and dissatisfaction and low self-regard with a conceivable outrageous result being burnout.

Physical strain is the second major strain caused by exposure to stressors. It is also known as physical health. Physical or physiological strain is theorized to appear in indications, for example, hypertension, abnormalities in blood eosinophils, and raised serum cholesterol [14]. Stress has been physically related to cardiovascular disorder, ulcers, hypertension, asthma, and headache cerebral agonies. Generally, investigators have a tendency to concur what the major physical strains brought on by stress are dysphoria, sleeping disorder and restlessness [17]. Physiological indicators are; heart illness, psychosomatic ailment, fatigue and depleted energy reserves. Occupational stress is supposed to assume a critical part in bringing on cardiovascular, gastrointestinal and musculoskeletal disorders [18]. Physical exhaustion may occur in the form of headache, shaking, incapability to think clearly and relax, lack of natural communication, anger resulting in short-tempered talk, vulnerability to common cold, cancer automotive diseases and experience of gastrointestinal problems. Stress can cause chronic fatigue, risk of stroke, worsen an asthma attack, proneness to accidents and athletic injuries [19].

The third characterization of strain is behavioral strain. Behavioral modifications are among the most effortlessly and effectively perceived indications of stress increasing [17]. Research revealed that increased cigarette smoking, increased alcohol and recreational medication abuse, hesitating, violence, overeating and regular visits of healthcare services are the symptoms of behavioral strain. Not all behavioral reactions to stressors ought to be organized as strain reactions, and only those reactions that are particularly and specifically dangerous to the individuals are the strain reactions [20]. Behavioral problems are, for example, craving issue, exorbitant smoking and liquor failure to rest, and possible displays of withdrawal indications (i.e. absenteeism and resignations from the employment).

The article "Relationship between perceived occupational stress and psychological well-being among secondary school heads in Khyber Pakhtunkhwa, Pakistan" was retracted in 2025. Reasons: duplicated data; duplicated text; overlap with earlier publications; unreliable data.

### Model of occupational stress

#### The person–environment fit model

The Person-Environment Fit Theory (P-E Fit Theory) was introduced by French, Rose, and Blackmore [21]. It is one of the most primitive supported conceptual models regarding job stress. It is a comprehensive idea that essentially consists of one's compatibility with numerous frameworks in occupational environment [22]. P-E fit refers to a compatibility between an individual's capabilities and the necessities of occupation. The key evidence of the theory is that stress emerges from the fit or consistency with the individual and environment and not from the individual or the environment disjointedly [21]. It proposes that unsatisfactory fit may contribute to physiological stress or mental stress or both. People are more successful, powerful, more fulfilled and more dedicated to their employments when their own characteristics match the characteristics of their situational surroundings. Research about the person-environment has been condemned fundamentally for lack of conceptualization of the environmental element of fit [22].

#### The job characteristics model

Job Characteristics Model emphasizes on the crucial aspects of job characteristics. For example, expertise assortment (what number of various aptitudes are required) task identity (how well usual functionalities are linked to overall work goals), task significance (how important the employment is), autonomy (how free the individual is to deal with their own working), and feedback (the amount of reward, commendation, or remarks the employee receives). These characteristics are endorsed to contribute to Critical Psychological States' of experienced importance, experienced obligation with respect to results, and information of employment outcomes. These characteristics may be positive or negative values. Positive attributes boost the mental states contributing to scholarly and behavioural outcomes e.g. satisfaction, inspiration, low level of absenteeism, sufficiency, productivity, advancement, turnover and so on. In conjunction with the model, Hackman and Oldham designed the Job Diagnostic Survey, a questionnaire for determining one's occupation, the outcomes of which propose five principal sorts of employment redesign: development of working units; joining assignments; making feedback techniques; making a client centered structure; and employment advancement [23].

The article "Relationship between perceived occupational stress and psychological well-being among secondary school heads in Khyber Pakhtunkhwa, Pakistan" was retracted in 2025. Reasons: duplicated data; duplicated text; overlap with earlier publications; unreliable data.

#### Effort reward imbalance model (ERI)

Effort Reward Imbalance (ERI) was introduced with aim to focus on cardiovascular disorders. The main idea of this model is one of reciprocity, or work as a component of a social change process. Echoing the balance orientation of the P-E fit model where a misfit between an individual's capabilities and the essentials of his employment causes strain, the important supposition of ERI is that efforts at work ought to be compensated by appropriate compensation, and a discrepancy between these will contribute to upsetting and distressing occurrences [21]. A condition which is specifically to be anticipated when an individual gets low rewards because of high efforts. Rewards are referred to career opportunities, money, respects and security. Effort is composed of two components i.e., intrinsic efforts and extrinsic inspirations. Intrinsic efforts take place from the personal motivation of an individual e.g., a need for control and over commitment (an inclination to make exceptional efforts or be dedicated on unpractical objectives). Extrinsic inspirations, or external pressures i.e., workload. ERI does not give a comprehensive redesign theory, yet like the DCS model, it supposes primary design principles in the light of essential interventions only, i.e. reasonable reward for effort, constructive criticism frameworks, and additional rewards and advancement prospects and so forth [24].

#### Job demand-control model

The Job Demands-Control Model was designed by Karasek based upon the supposition that the relationship between employment demands and employment control will describe strain consequences [25]. Job demand is defined as the independent variable that gauges stressors, for example, workload demands. Job control was initially conceptualized under the expression job decision latitude and characterized it as a control that the working personnel has completed tasks and their execution during their functioning day. Karasek recommended that when employment demands are high than employment control, strain will take place, contributing to both psychological and physical health issues [25]. The idea of job control has for quite some time been recognized as a vital factor in the process of occupational stress, but a question arises that how to operationalize this model and how the relationship between demands and control ought to be measured have contributed to conflicting findings and trouble in replicating Karasek’s proposed model [26]. Job Demand-Control Model classifies jobs into four kinds in the light of various blends of demands and control. The primary sort called "active" and happens when the workforces have high demands and high control in the meantime. Alternately, the second sort called "passive" and takes place when the workforces encounter little demands and they do not need high control. The third sort called "relaxed" and takes place when the workers encounter little demands and they have high control. The fourth kind which is the most stressful and upsetting situation called "Job strain" and occurs when the workforces experience too high demands while they have little control to deal with over-burden, conflict, ambiguities and stress [25].

The article "Relationship between perceived occupational stress and psychological well-being among secondary school heads in Khyber Pakhtunkhwa, Pakistan" was retracted in 2025. Reasons: duplicated data; duplicated text; overlap with earlier publications; unreliable data.

#### Job-demands-resources model

Job-Demands-Resources Model is one of the prominent models of occupational stress [26] and is linked to the Burnout Model [27]. Continuous stress is emotionally depleting and eventually prompts to a condition of 'burnout'. Burnout has been conceptualized as a mental disorder created because of interminable interpersonal stressors at work and is described by three key measurements. Firstly, burnout is described by incontrollable exhaustion, secondly by emotions of cynicism and separation from the employment, lastly by a feeling of incapability and lack of accomplishment. The exhaustion component denotes the stress dimensions of burnout, that the cynicism component describes the interpersonal context of burnout, and that the incapability and lack of accomplishment components describe the self-evaluation dimension of burnout [27]. This model suggests that the two processes are responsible for the development of burnout. Firstly, intense employment demands prompt to consistent straining of the individual and, ultimately to emotional exhaustion. Secondly, inadequate resources accessible to the workers confounds the fulfilling of employment demands which then contribute to withdrawal behaviours and finally to discontinuation of work. The Job-Demands-Resources Model accepts that despite the fact that workers in various associations might be gone up against with various working conditions, the characteristics of these working conditions can be ordered into two classifications–job demands and job resources. Job resources are characterized as similar parts of one's employment (physical, mental, social or organizational) but those parts are useful in accomplishing work objectives, diminishing employment demands, or animating self-improvement and development. Like the models of occupational stress introduced over, the Job-Demands-Resources Model deals with the supposition that stress in the working environment is caused due to interaction between individual and their surroundings [28].

The article "Relationship between perceived occupational stress and psychological well-being among secondary school heads in Khyber Pakhtunkhwa, Pakistan" was retracted in 2025. Reasons: duplicated data; duplicated text; overlap with earlier publications; unreliable data.

#### Transactional theory of stress and coping

The Transactional Theory of Stress and Coping was presented by Lazarus and Folkman [29]. This model stresses the progressing and the mutual collaboration between the individual and the environment. In view of this theory, stress is not occurred in individual or condition independently, however in the connection between the condition of people's appraisal of the working and ceaseless attempts to manage issues that develop [30]. In this theory, two processes distinguished the association between the individual and environment. In the first process “cognitive appraisal”, one assesses the significance and effect of a specific experience with the environment to the prosperity of the individual. This includes evaluation of potential stressors as undermining and representing some sort of risk to the person. Cognitive appraisal is proposed to assume a vital role in the coping process. As the working environment is continuously changing, individuals observe diverse distressing circumstances in various ways and differ their utilization of adapting techniques crosswise over upsetting circumstances. This implies that flexible stress appraisal encourages flexible coping responses [31]. The second process "coping" accomplishes certain internal and external requirements that are subjected to measure as stimulating and surpassing one's resources by changing cognitive and behavioral efforts [29]. This includes the assessment of coping resources and alternate reactions. If a man sees that a circumstance is undermining, but can cope it, then trouble is not faced and this circumstance is seen as interesting and challenging. In this model, coping is viewed as a vital technique on how people associate with the circumstances and is a continuous developing process that happens within the line of modifying people and situational demands [31]. Likewise, Folkman and Moskowitz [32] has characterized coping as the thoughts and behaviours utilized by people to control both the internal as well as external demands of conditions which are assessed as unpleasant. Wilhelm et al. [33] found that some people have a tendency to change their methods of coping in various circumstances, while others tend to utilize similar courses regardless of situational characteristics.

A difference is normally created between problem focused coping that resolves the demands of a stressor while emotion focused coping assists the individual to feel better about the stressor [29]. Stress and problems emerge when a man assesses the demands of a circumstance as going to surpass the existing resources and to be a risk for his/her prosperity, demanding an adjustment in individual working to return balance [34]. Fickova [35] expressed that affectivity (positive and negative) indicates that which coping technique to be operated at the time of upsetting and distressing circumstances. If feelings were rigorous, they modify the nature of the data processing approach and understanding to the individual that something is not right. Furthermore, if feelings were of low strength, they indicate that all is going well. Folkman and Lazarus [36] summarized the process in this model. A potentially distressing occasion will produce the primary appraisal process in which a man assesses the degree of danger in connection to his/her prosperity. When an occasion is seen as aggressive or a challenging, the secondary appraisal process gives a worldwide assessment of the individual's coping resources and capability to deal with the risk and challenge. Coping responses begin after the cognitive appraisals and the stress consequences of this potentially upsetting occasion depend on the competency of one's cognitive appraisals and coping processes. In spite of the fact that the transactional theory can anticipate individual contrasts in the experience and response to stress, it cannot foresee which facets of the workplace will be distressing [31]. The transactional theory of stress and adapting system is the most suitable on account of its flexibility and mental enquiry about convictions, perspectives and practices related stress. Besides, the transactional model has a few qualities; it clarifies adapting in steps, underlines the significance of thinking, recognition, and assurance of controllability, accentuates the role of ceaseless stressors or day by day disturbances as being more essential than every so often life occasions; tracks into account the association amongst individual and environment; and has a feedback system in the form of assessment or appraisal [37].

The article "Relationship between perceived occupational stress and psychological well-being among secondary school heads in Khyber Pakhtunkhwa, Pakistan" was retracted in 2025. Reasons: duplicated data; duplicated text; overlap with earlier publications; unreliable data.

### Psychological well-being

The significance of psychological well-being at work has been recognized in the last few decades as there has been a move from physical to psychological wellsprings of pressure at work. From various perspectives, pressure at work is psychologically healthy. It gives individuals a chance to experience a feeling of challenge and accomplishment, both of which are crucial for high level of psychological well-being. However, when pressures turn out to be excessively troublesome or frequent to deal with, psychological well-being is badly affected rather than improved [38]. Well-being has turned into a mainstream point in logical research as it is seen by numerous authors as imperative to workers’ overall wellbeing and advancement since it incorporates an all-encompassing viewpoint of individual health [39]. Well-being refers to the experience of meaning, attitudes, behaviours, social connections and the individual's interconnectedness with the environment [40]. Wright [41] defines psychological well-being as, a subjective and worldwide judgment that one is encountering a maximal positive and generally minimal negative emotions or feelings. Psychological well-being is the capability of an individual to feel satisfied and perform effectively regardless of negative or throbbing feelings which are typically part of life [42]. According to Chaturvedula and Joseph [43], psychological well-being is a man's judgment or assessment of his or her life–either regarding life fulfillment (intellectual assessments) or influence (emotional reactions) which is additionally partitioned into pleasant effect (positive emotions) and unpleasant effect (negative emotions). Moe [44] considers psychological well-being as the foundation stone of emotional wellness. Psychological well-being is simply defined as ultimately about individual satisfaction—feeling good and living safely and healthily. Psychological well-being is composed of all the short-term and long-term mental functioning and positive well-being (e.g. positive affect, self-confidence and morale) and negative well-being (e.g. depression, discouragement, anxiety) [45].

Organizational productivity and efficiency depends on the employees’ satisfaction, happiness and good wellbeing [46]. Psychological well-being has to do with people’s feeling in the routine life, and these feelings may vary from positive feelings i.e., satisfaction, happiness etc to negative feelings i.e., depression and dissatisfaction. Psychological well-being is composed of our capability to deal with stress in day-to-day life through positive attitudes and purpose of life. It has been proved by research that psychological well-being has connection to success and health [47]. Organizations where employees’ psychological well-being is healthy are achieving productive outcomes and even employees having high psychological well-being are enthusiastic to come to work. Conversely, employees having low psychological well-being will exhibit absenteeism. Individual respect if they have independence in functioning, they are involved in decision making and there is no unrealistic workload pressure. Employees wish to be safe, valuable and satisfied in their working environment [48]. Enhancing the employees’ psychological well-being brings benefits for them as well as for organization. Psychological well-being is the fundamental component of overall well-being and is related to physical well-being, longer lives and greater pleasure for employees [38]. Psychological well-being of the employees has a link with organizational productivity and efficiency. Satisfactory and good work provides opportunities to employees for promoting their well-being and prosperity [49]. Shagvaliyeva and Yazdanifard [50] expressed that employees’ mental, physical and personal well-being may affect their performance and productivity. Mental well-being is a critical indicator of a happy and healthy life. Mentally sickened employees will exhibit poor and undesirable behaviour at work and personal domain. Occupational stress causes depression and anxiety as a result of unsatisfactory employees’ performance. Long-term and exorbitant stress can be a serious danger for employees’ well-being.

The article "Relationship between perceived occupational stress and psychological well-being among secondary school heads in Khyber Pakhtunkhwa, Pakistan" was retracted in 2025. Reasons: duplicated data; duplicated text; overlap with earlier publications; unreliable data.

### Review of relevant research studies

A number of research studies have been conducted on the relationship between occupational stress and psychological well-being in different fields. Malek, Fahrudin and Kamil [51] led an investigation on the sources of occupational stress and their impact on job satisfaction and psychological well-being. They found a significant reverse relationship between the sources of occupational stress and job satisfaction as well as well-being. Yunus and Mahajar [52] carried out a research study on stress and psychological well-being of government officers in Malaysia and they found that four dimensions of occupational stress i.e., role overload, role insufficiency, role ambiguity and role boundary have substantial relationship and impact on psychological well-being. Adegoke [53] analyzed the effects of occupational stress on psychological well-being of police employees and found that there was significant effect of work-stress, depression and frustration on psychological well-being of police employees in Ibadan metropolis. Khan and Khurshid [54] investigated the impact of workplace stress on employees’ well-being in the medicinal sector and hospitals in UAE. They found that working environment has a negative impact on employees’ well-being and the impact was found to be weak. They concluded that stressful working environment will reduce employees’ well-being. Poormahmood, Moayedi, and Alizadeh [55] conducted a cross-sectional study on the relationship between psychological well-being, happiness and perceived occupational stress among primary school teachers and found negative correlation between occupational stress and four subscales of psychological well-being i.e., life satisfaction, spirituality, joy and optimism, individual development while positive correlation with relationships with others, and autonomy, as well as with overall psychological well-being. They concluded that occupational stress in teaching may lead to poor psychological well-being and reduced happiness in primary school teachers.

The article "Relationship between perceived occupational stress and psychological well-being among secondary school heads in Khyber Pakhtunkhwa, Pakistan" was retracted in 2025. Reasons: duplicated data; duplicated text; overlap with earlier publications; unreliable data.

## Objectives of the study

The purpose of the study was to examine the relationship between perceived occupational stress and psychological wellbeing among secondary school heads in Khyber Pakhtunkhwa, Pakistan. The objectives of the study were:

1. To examine the relationship between perceived occupational stress and psychological well-being among secondary school heads in Khyber Pakhtunkhwa
2. To establish the contribution of each dimension of occupational stress in predicting the psychological well-being among secondary school heads in Khyber Pakhtunkhwa

## Hypotheses of the study

**Hypothesis 1.** *There is no significant relationship between perceived occupational stress and psychological well-being among secondary school heads*.

**Hypothesis 2.** *There is no significant relationship between the subscales of perceived occupational stress and psychological well-being among secondary school heads*.

**Hypothesis 3.** *Subscales of perceived occupational stress have no significant contribution in predicting psychological well-being among secondary school heads*.

## Methods and materials

### Study population

The study was conducted in the province of Khyber Pakhtunkhwa (Pakistan) which is located in the north-western region of the country. It is divided into seven divisions and 25 districts. Peshawar is the largest city and provincial capital of Khyber Pakhtunkhwa. It was previously recognized by North-West Frontier Province (NWFP). The study in hand was conducted in 10 out of 25 districts of Khyber Pakhtunkhwa namely, Karak, Kohat, Hangu, Peshawar, Bannu, Abbottabad, Nowshera, Charssada, Lakki Marwat, and Malakand. In educational research, it is imperative to ensure an accurate depiction of the population of the subjects or elements under investigation i.e., persons, objects, organizations etc. The entire group of individuals to which the investigator generalizes the results is called population. In current study, all the secondary school heads in Khyber Pakhtunkhwa constituted the population of the study. In the light of EMIS Report published by Education Department of Khyber Pakhtunkhwa, there were total 2108 functional public secondary schools in Khyber Pakhtunkhwa (Male *n* = 1386; Female *n* = 722). The total number of secondary school heads in these schools were 2108 (Male *n* = 1386; Female *n* = 722) (see Table 1) [56].

**Table 1:** Population and sample size of the study.

S. No.	Districts	No. of Schools				No. of Heads			
		Total		Sample		Total		Sample	
		Male	Female	Male	Female	Male	Female	Male	Female
1.	Karak	56	26	37	16	37	16	28	12
2.	Peshawar	85	55	51	33	51	33	38	25
3.	Kohat	47	27	28	16	28	16	21	12
4.	Bannu	59	40	35	24	35	24	26	18
5.	Abbottabad	69	45	41	27	41	27	31	20
6.	Nowshera	66	29	40	17	40	17	30	13
7.	Hangu	26	09	16	05	16	05	12	04
8.	Lakki Marwat	56	21	34	13	34	13	26	10
9.	Charssadda	61	33	37	20	37	20	28	15
10.	Malakand	45	29	27	17	27	17	20	13
**Total**		**570**	**314**	**346**	**188**	**346**	**188**	**260**	**142**

The article "Relationship between perceived occupational stress and psychological well-being among secondary school heads in Khyber Pakhtunkhwa, Pakistan" was retracted in 2025. Reasons: duplicated data; duplicated text; overlap with earlier publications; unreliable data.

### Sample and sampling techniques

In educational research, multi-stage sampling technique is extensively practiced globally as it is more systematic, convenient and trustworthy. Multistage sampling is used when the population is widely scattered and adequate resources are not available. Different sampling techniques may be used for selecting sample at each stage according to the nature of the population i.e., simple random sampling technique, stratified sampling technique etc. Simple random sampling is the simplest of the probability sampling techniques. A complete sampling frame is required for such sampling technique which is difficult to construct for larger populations. A simple random sample is a sample selected in such a way that every possible sample of the same size is equally expected to be selected. On the other hand, stratified sampling is used when the population may heterogeneous due to some characteristics i.e., gender, locality, income level, educational level etc. It refers to the breakdown of the population into homogeneous and non-overlapping groups (i.e., strata) and after stratification of the population, simple random sampling is used to generate the entire sample. In current study, the population was widely scattered and it was not possible to select sample randomly. So, multistage sampling was adopted for selecting sample. According to Gay [57], if the population had around 500 subjects, then 50% of the subjects may be sampled. If the size of the population is 1,500, then the sample should be taken 20%. Beyond a certain point (at approx. N = 5,000), a sample size of 400 will be sufficient. Hence, a researcher needs to take sample at smaller percentage if the population is larger. Additionally, Gay and Diehl [58] expressed that sample comprised of 10% of the population is adequate for a descriptive research. However, if the population size is small then 20% should be taken. On the other hand, in correlational research, at least 30 subjects are sufficient to examine a relationship between the variables. But for the sake of validation of the findings, in current study, adequate sample size was taken. So, at first stage 10 (40%) out of 25 districts of Khyber Pakhtunkhwa i.e., Kohat, Karak, Bannu, Abbottabad, Peshawar, Lakki Marwat, Nowshera, Charssada, Malakand and Hangu were carefully chosen randomly as a primary sampling unit. At second stage, 60% Boys and 60% Girls secondary schools were selected with the help of stratified sampling technique as secondary sampling unit. At third stage, 75% male and 75% female secondary school heads were selected randomly from the said selected secondary schools as tertiary sampling unit. In this way, the total sample comprised of 402 secondary school heads (Male *n* = 260; Female *n* = 142) selected from 534 government secondary schools located in the sample districts (See Fig 1). Table 1 shows the population and sample size of the study.

The article "Relationship between perceived occupational stress and psychological well-being among secondary school heads in Khyber Pakhtunkhwa, Pakistan" was retracted in 2025. Reasons: duplicated data; duplicated text; overlap with earlier publications; unreliable data.

**Fig 1:** Multistage sampling technique.

### Measurements

The study was aimed to examine the relationship between perceived occupational stress and psychological well-being among secondary school heads in Khyber Pakhtunkhwa. For this purpose, two measuring tools i.e., Occupational Stress Index (OSI) and Ryff’s Psychological Well Being Scale (RPWB) were utilized for gathering information from the participants after taking formal permission from their authors. Each tool has been explained in detail as under:

#### Occupational stress index (OSI)

The occupational stress was measured through Occupational Stress Index (OSI) originally designed and standardized by Shrivatsava and Singh [59]. OSI is a widely acceptable scale for measuring job stress. It has been applied by a number of psychologists in researches. The scale is specially designed to measure the stress which is perceived by the workforce from numerous conditions and dimensions of their job position. The scale may be used to assess the stress of the workforces employed in context of industries or other non-production departments such as, education, medical etc. The scale consists of twelve dimensions i.e., role overload, role conflict, role ambiguity, unreasonable group & political pressure, under participation, responsibility for persons, powerlessness, intrinsic impovishment, peer group relations, low status, strenuous working condition, and unprofitability (See S1 Appendix). The scale comprises of 46 items designed on five-point likert scale. Among these items, 28 were true keyed and 18 were false keyed items. The true keyed items were rated as 5 = strongly agree, 4 = agree, 3 = undecided, 2 = disagree and 1 = strongly disagree while the false keyed items were rated as reversed. The reliability coefficient calculated by Split Half (odd-even) strategy and Cronbach's Alpha Coefficient for the scales were found to be 0.937 and 0.90 respectively.

The article "Relationship between perceived occupational stress and psychological well-being among secondary school heads in Khyber Pakhtunkhwa, Pakistan" was retracted in 2025. Reasons: duplicated data; duplicated text; overlap with earlier publications; unreliable data.

Occupational Stress Index (OSI) is highly reliable standardized research instrument which is used to gauge occupational stress of the employees in different context. In the light of social and culture context, it was important to confirm its reliability and therefore Cronbach’s Alpha was used to calculate the reliability of OSI. Table 2 shows the Average Internal Consistency Reliability (Cronbach’s Alpha) of the subscales of Occupational Stress Index (OSI). Cronbach’s Alpha shows that each subscale has a high reliability coefficient. Additionally, the analysis reveals that the overall internal consistency reliability (Cronbach’s Alpha) of OSI was computed as 0.872 which confirms that OSI is exceptionally reliable research instrument for measuring occupational stress.

**Table 2:** Average internal consistency reliability (cronbach’s alpha) of the sub-scales of occupational stress index (OSI).

**Sub-Scales of OSI**	**No. of Items**	**Cronbach’s α Coefficient**
Role Overload	06	0.887
Role Ambiguity	04	0.846
Role Conflict	05	0.896
Unreasonable Group & Political Pressure	04	0.788
Responsibility for Persons	03	0.844
Under Participation	04	0.869
Powerlessness	03	0.986
Peer Group Relations	04	0.854
Intrinsic Impoverishment	04	0.786
Low Status	03	0.877
Strenuous Working Conditions	04	0.838
Unprofitability	02	0.998
**Mean**	**3.83**	**0.872**

#### Ryff’s psychological wellbeing scale (RPWB)

In order to measure psychological wellbeing of the research participants, Psychological Wellbeing Scale (RPWB) developed by Ryff [60] was used. The scale is composed of self-reported 42 items and includes six domains i.e., autonomy, environmental mastery, personal growth, positive relations with others, purpose of life, and self-acceptance (See S2 Appendix). Each domain has seven items and the responses were documented by means of a 6-point Likert scale ranging from 1 = strongly disagree to 6 = strongly agree. Among these items, 47 items were scored as 6 = strongly agree to 1 = strongly disagree and the rest of the items were scored reversed due to their negative nature. The higher scores indicate greater experience of psychological well-being and positive effects. Although the scale has high validity and reliability but it was imperative to check its validity and reliability in the current study population. That’s why it was validated through five experts. Cronbach’s Alpha was used to calculate the reliability of Ryff’s Psychological Wellbeing Scale (RPWB). Table 3 indicates the Average Internal Consistency Reliability (Cronbach’s Alpha) of each domain of the scale. Cronbach’s Alpha shows that each subscale has a high reliability coefficient. Additionally, the analysis reveals that the overall internal consistency reliability (Cronbach’s Alpha) of RPWB was found 0.784 which confirms that RPWB is highly reliable research instrument for measuring psychological wellbeing.

The article "Relationship between perceived occupational stress and psychological well-being among secondary school heads in Khyber Pakhtunkhwa, Pakistan" was retracted in 2025. Reasons: duplicated data; duplicated text; overlap with earlier publications; unreliable data.

**Table 3:** Average internal consistency reliability (cronbach’s alpha) of the sub-scales of ryff’s psychological wellbeing scale (RPWB).

Subscales of (RPWB) Scale	No. of Items	Cronbach’s α Coefficient
Autonomy	07	0.793
Environmental Mastery	07	0.776
Personal Growth	07	0.836
Positive Relations with Others	07	0.778
Purpose of Life	07	0.777
Self-Acceptance	07	0.744
**Mean**	**07**	**0.784**

### Data collection and analysis

Before the commencement of research study, it was approved by the Advance Studies & Research Board (ASRB) of Kohat University of Science & Technology (Pakistan). After the approval of the study from ASRB, it was imperative to seek the permission from the Director of Elementary & Secondary Education Khyber Pakhtunkhwa, Pakistan. So, after getting formal permission (See S3 Appendix) from the Director, data collection process was commenced on November 15, 2016 and completed on February 15, 2017. In some of the districts, data were collected through personal visits. However, data was also collected through mail in case of far-flung areas. For this purpose, questionnaires were mailed to participants on their school addresses in six districts of Khyber Pakhtunkhwa i.e., Peshawar, Malakand, Charssadda, Nowshera, Bannu and Abbottabad. Participants were provided with a covering letter explaining the purpose of the study. In covering letter, the participants were told that completion of the questionnaires would be considered to be their consent to participate in the study. They were also informed that their responses would be kept confidential and would be used only for the research purposes. Additionally, they were assured that their responses would be destroyed immediately after analyzing the data. In addition to covering letter, a self-addressed envelope was enclosed with each mailing registered letter for returning the questionnaires after completion. To get maximum response rate, follow-up study was done. Due to follow-up study, 100% responses were received successfully. Statistical Analysis was done through SPSS version 25. Demographic characteristics were presented through simple percentage. Statistical tools i.e., mean, standard deviation, Pearson’s Product Moment Correlation and Multiple Linear Regression were performed to achieve the research objectives.

## Results

### Participants’ demographic characteristics

In this study, 402 secondary school heads (male *n* = 260, female *n* = 142) participated on the request of researchers through formal permission. As presented in Table 4, the statistical analysis indicates that 64.68% secondary school heads were males and 35.32% were females. In case of age, 6.71% secondary school heads were in age group 30–34 years, 12.19% were in age group 35–39 years, 18.90% were in age group 40–44 years and 62.19% were in age group 45 years & above. In term of service length, 46.77% heads had (01–04) years, 25.62% had (05–09) years, 17.16% had (10–14) years, and 10.45% had 15 years & above. In terms of academic educational level, 46 (11.44%) were bachelor degree holders, 341 (84.83%) were Master degree holders, 12 (02.99%) were M.Phil degree holders and 03 (00.75%) were PhD degree holders. In case of professional qualification, 221 (54.98%) were bachelor degree holders, 168 (41.79%) were Master degree holders, 11 (02.74%) 02 (00.50%) were M.Phil degree holders and 03 (00.75%) were PhD degree holders. With respect to locality, 90 (22.39%) heads belonged to urban localities while 312 (77.61%) heads belonged to rural localities.

The article "Relationship between perceived occupational stress and psychological well-being among secondary school heads in Khyber Pakhtunkhwa, Pakistan" was retracted in 2025. Reasons: duplicated data; duplicated text; overlap with earlier publications; unreliable data.

**Table 4:** Descriptive statistics of demographic information of secondary school heads (n = 402).

Variables	Categories	n (%)
Gender	Male	260 (64.68%)
	Female	142 (35.32%)
Age (in years)	30–34	27 (06.715%)
	35–39	49 (12.19%)
	40–44	76 (18.90%)
	45 & Above	250 (62.19%)
Experience (in years)	01–04	188 (46.77%)
	05–09	103 (25.62%)
	10–14	69 (17.16%)
	15 & above	42 (10.45%)
Academic Qualification	B.A	46 (11.44%)
	M.A	341 (84.83%)
	M.Phil	12 (02.99%)
	Ph.D	03 (00.75%)
Professional Qualification	B.Ed	221 (54.98%)
	M.Ed	168 (41.79%)
	M.Phil (Edu)	11 (02.74%)
	Ph.D (Edu)	02 (00.50%)
Locality	Urban	90 (22.39%)
	Rural	312 (77.61%)

### Descriptive statistics

#### Perceived occupational stress

Table 5 presents the descriptive statistics of the occupational stress among secondary school heads. The results revealed that the most rated subscale of occupational stress was role overload (*X = 3*.*55*, *SD = 0*.*675*) followed by unprofitability (*X = 3*.*53*, *SD = 0*.*900*). The other subscales of occupational stress were rated as unreasonable group and political pressure (*X = 3*.*52*, *SD = 0*.*721*), strenuous working condition (*X = 3*.*48*, *SD = 0*.*748*), powerlessness (*X = 3*.*41*, *SD = 0*.*954*), and role conflict (*X = 3*.*39*, *SD = 0*.*803*), under participation (*X = 3*.*33*, *SD = 0*.*834*). It clearly shows that secondary school heads were occupationally stressed with these dimensions of occupational stress. Furthermore, it was found that secondary school heads were not occupationally stressed with respect to responsibility for persons (*X = 2*.*94*, *SD = 0*.*999*), low status (*X = 2*.*63*, *SD = 0*.*703*), peer group relations (*X = 2*.*46*, *SD = 0*.*711*), role ambiguity (*X = 2*.*42*, *SD = 0*.*661*), and intrinsic impoverishment (*X = 2*.*40*, *SD = 0*.*618*).

The article "Relationship between perceived occupational stress and psychological well-being among secondary school heads in Khyber Pakhtunkhwa, Pakistan" was retracted in 2025. Reasons: duplicated data; duplicated text; overlap with earlier publications; unreliable data.

**Table 5:** Descriptive statistics of the perceived occupational stress among secondary school heads (n = 402).

Variables	Min	Max	Mean±SD	SE	Skewness		Kurtosis	
					Statistic	SE	Statistic	SE
ROL	1.50	5.00	3.55±0.675	.03364	-.147	.122	.261	.243
RA	1.00	4.50	2.42±0.661	.03295	.391	.122	-.169	.243
RC	1.20	5.00	3.39±0.803	.04005	-.032	.122	-.432	.243
UGPP	1.25	5.00	3.52±0.721	.03595	-.119	.122	-.012	.243
RP	1.00	5.00	2.94±0.999	.04984	-.103	.122	-.994	.243
UP	1.00	5.00	3.33±0.834	.04158	-.183	.122	-.189	.243
P	1.00	5.00	3.41±0.954	.04756	-.216	.122	-.619	.243
PGR	1.00	5.00	2.46±0.711	.03548	.417	.122	.009	.243
II	1.00	4.50	2.40±0.618	.03085	.649	.122	.652	.243
LS	1.00	5.00	2.63±0.703	.03506	.332	.122	-.335	.243
SWC	1.25	5.00	3.48±0.748	.03732	-.206	.122	-.194	.243
U	1.00	5.00	3.53±0.900	.04487	-.146	.122	-.521	.243

Key: ROL = Role Overload; RA = Role Ambiguity; RC = Role Conflict; UGPP = Unreasonable Group & Political Pressure; RP = Responsibility for Persons; UP = Under Participation; P = Powerlessness; PGR = Peer Group Relation; II = Intrinsic Improvishment; LS = Low Status; SWC = Strenuous Working Conditions; U = Unprofitability; PWB = Psychological Well-being

#### Psychological well-being

Table 6 portrays the descriptive statistics of the psychological well-being among secondary school heads. The outcomes of the descriptive analysis revealed that the most rated subscale of psychological well-being was positive relations with others (*X = 4*.*34*, *SD = 0*.*333*) followed by self-acceptance (*X = 4*.*30*, *SD = 0*.*349*). The other subscales of psychological well-being were rated as environmental mastery (*X = 4*.*29*, *SD = 0*.*380*), purpose of life (*X = 4*.*29*, *SD = 0*.*334*), autonomy (*X = 4*.*22*, *SD = 0*.*416*), and personal growth (*X = 4*.*20*, *SD = 0*.*360*). It clearly indicates that secondary school heads possess good psychological well-being.

**Table 6:** Descriptive statistics of the psychological well-being among secondary school heads (n = 402).

Variables	Min	Max	Mean±SD	SE	Skewness		Kurtosis	
					Statistic	SE	Statistic	SE
A	3.02	4.97	4.22±0.416	0.021	-.355	.122	-.456	.243
EM	3.04	4.99	4.29±0.380	0.019	-.480	.122	.347	.243
PG	3.14	5.21	4.20±0.360	0.018	-.387	.122	-.221	.243
PRO	3.17	4.98	4.34±0.333	0.017	-.625	.122	.347	.243
PL	3.32	4.96	4.27±0.334	0.017	-.688	.122	.228	.243
SL	3.17	4.96	4.30±0.349	0.017	-.594	.122	.058	.243

Key: A = Autonomy, EM = Environmental Mastery, PG = Personal Growth, PRO = Positive Relations with Others, PL = Purpose of Life, SA = Self-Acceptance

The article "Relationship between perceived occupational stress and psychological well-being among secondary school heads in Khyber Pakhtunkhwa, Pakistan" was retracted in 2025. Reasons: duplicated data; duplicated text; overlap with earlier publications; unreliable data.

### Pearson’s Correlation/Multiple linear regression analysis

#### Hypothesis 1

*There is no significant relationship between perceived occupational stress and psychological well-being among secondary school heads*.

In order to find out the correlation between perceived occupational stress and psychological well-being, Pearson’s product moment correlation was performed. According to the results of Table 7, there is a strong negative correlation (*r = -0*.*947*, *p<0*.*01*) between perceived occupational stress and psychological well-being. It means that perceived occupational stress has negative impact on phycological well-being. An occupationally stressed head will have a poor psychological well-being in workplace. Hence the null hypothesis “there is no significant relationship between perceived occupational stress and psychological well-being among secondary school heads” was rejected.

**Table 7:** Pearson’s product-moment correlation analysis between perceived occupational stress and psychological well-being among secondary school heads (n = 402).

Variables		POS	PWB
**POS**	Pearson Correlation	1.00	-.947**
	Sig. (2-tailed)	-	.000
	N	402	402
**PWB**	Pearson Correlation	-.947**	1.00
	Sig. (2-tailed)	.000	-
	N	402	402

** Correlation is significant at the 0.01 level (2-tailed).

Correlation Strength: r ≥ 0.70 = Strong; 0.30 ≤ r ≤ 0.69 = Moderate; 0.01 ≤ r ≤ 0.29 = Weak

Key: POS = Perceived Occupational Stress; PWB = Psychological Well-being

#### Hypothesis 2

*There is no significant relationship between the subscales of perceived occupational stress and psychological well-being among secondary school heads*.

Pearson’ correlation was applied to examine the correlation between the dimensions of occupational stress and psychological well-being among secondary school heads. As Table 8 indicates, a moderate negative correlation was found between all the dimensions of perceived occupational stress and psychological well-being i.e., role overload (*r = -0*.*653*, *p<0*.*01*), role ambiguity (*r = -0*.*464*, *p<0*.*01*), role conflict (*r = -0*.*646*, *p<0*.*01*), unreasonable group & political pressure (*r = -0*.*598*, *p<0*.*01*), responsibility for persons (*r = -0*.*309*, *p<0*.*01*), under participation (*r = -0*.*624*, *p<0*.*01*), powerlessness (*r = -0*.*601*, *p<0*.*01*), peer group relation (*r = -0*.*550*, *p<0*.*01*), intrinsic improvishment (*r = -0*.*495*, *p<0*.*01*), low status (*r = -0*.*614*, *p<0*.*01*), strenuous working conditions (*r = -0*.*642*, *p<0*.*01*), and unprofitability (*r = -0*.*554*, *p<0*.*01*). Hence, the null hypothesis “there is no significant correlation between the sub-scales of perceived occupational stress and psychological well-being among secondary school heads.” was rejected.

The article "Relationship between perceived occupational stress and psychological well-being among secondary school heads in Khyber Pakhtunkhwa, Pakistan" was retracted in 2025. Reasons: duplicated data; duplicated text; overlap with earlier publications; unreliable data.

**Table 8:** Pearson’s product-moment correlation (r) between the sub-scales of perceived occupational stress and psychological well-being among secondary school heads.

Variables	ROL	RA	RC	UGPP	RP	UP	P	PGR	II	LS	SWC	U	PWB
**ROL**	1.00												
**RA**	.196**	1.00											
**RC**	.483**	.318**	1.00										
**UGPP**	.543**	.169**	.500**	1.00									
**RP**	.199**	.085	-.044	.087	1.00								
**UP**	.421**	.195**	.613**	.436**	.025	1.00							
**P**	.405**	.269**	.276**	.309**	.085	.314**	1.00						
**PGR**	.223**	.300**	.245**	.134**	.171**	.330**	.321**	1.00					
**II**	.174**	.274**	.194**	.079	.117*	.290**	.248**	.848**	1.00				
**LS**	.423**	.295**	.293**	.324**	.087	.337**	.946**	.332**	.268**	1.00			
**SWC**	.515**	.268**	.594**	.516**	.093	.492**	.267**	.185**	.144**	.289**	1.00		
**U**	.479**	.130**	.426**	.470**	.091	.297**	.231**	.121*	.102*	.236**	.430**	1.00	
**PWB**	-.653**	-.466**	-.646**	-.598**	-.309**	-.624**	-.601**	-.550**	-.495**	-.614**	-.642**	-.554**	1.00

**. Correlation is significant at the 0.01 level (2-tailed)

*. Correlation is significant at the 0.05 level (2-tailed).

Correlation Strength: r ≥ 0.70 = Strong; 0.30 ≤ r ≤ 0.69 = Moderate; 0.01 ≤ r ≤ 0.29 = Weak

Key: ROL = Role Overload; RA = Role Ambiguity; RC = Role Conflict; UGPP = Unreasonable Group & Political Pressure; RP = Responsibility for Persons; UP = Under Participation; P = Powerlessness; PGR = Peer Group Relation; II = Intrinsic Improvishment; LS = Low Status; SWC = Strenuous Working Conditions; U = Unprofitability; PWB = Psychological Well-being

#### Hypothesis 3

*Subscales of perceived occupational stress have no significant contribution in predicting psychological well-being among secondary school heads*.

As presented in Table 9, a multiple regression analysis was performed to determine the contribution of each independent variable (subscales of perceived occupational stress) in predicting the dependent variable (psychological well-being). The model is statistically significant *(p = 0*.*000)* as the value of ANOVA was found to be 287.258 which is greater than the table value. Furthermore, the table indicates that the value of R square is 0.899 which shows that 90% of the variance in psychological well-being is significantly represented by the independent variables in the model. The results of regression analysis revealed that except low status (*β = -0*.*042*, *p>0*.*05*), all the subscales of occupational stress were found substantial predictors and have significant negative effect on psychological well-being i.e., role overload (*β = -0*.*091*, *p<0*.*05*), role ambiguity (*β = -0*.*140*, *p<0*.*05*), role conflict (*β = -0*.*137*, *p<0*.*05*), unreasonable group & political pressure (*β = -0*.*122*, *p<0*.*05*), responsibility for persons (*β = -0*.*186*, *p<0*.*05*), under participation (*β = -0*.*137*, *p<0*.*05*), powerlessness (*β = -0*.*203*, *p<0*.*05*), peer group relation (*β = -0*.*099*, *p<0*.*05*), intrinsic improvishment (*β = -0*.*159*, *p<0*.*05*), strenuous working conditions (*β = -0*.*148*, *p<0*.*05*), and unprofitability (*β = -0*.*170*, *p<0*.*05*). Hence, the null hypothesis “Subscales of perceived occupational stress have no significant contribution in predicting psychological well-being among secondary school heads.” was rejected. It plainly indicates that occupational stress has reverse relationship with psychological well-being and it can harm psychological well-being of the employees in workplace.

The article "Relationship between perceived occupational stress and psychological well-being among secondary school heads in Khyber Pakhtunkhwa, Pakistan" was retracted in 2025. Reasons: duplicated data; duplicated text; overlap with earlier publications; unreliable data.

**Table 9:** Multiple linear regression to analyse the contribution of each independent variable (dimensions of perceived occupational stress) in predicting the dependent variable (psychological well-being) among secondary school heads (n = 402).

Psychological Well-being (Dependent Variable)									
Model		Unstandardized Coefficients		Standardized Coefficients	*t*	*Sig*.	*R* Square	*F*	*Sig*.
		*B*	Std. Error	*β*					
Independent Variables	(Constant)	5.544	.023		236.161	.000	0.899	287.258	0.000
	ROL	-.027	.007	-.091*	-4.087	.000			
	RA	-.038	.005	-.140*	-7.746	.000			
	RC	-.032	.006	-.137*	-5.617	.000			
	UGPP	-.033	.006	-.122*	-5.696	.000			
	RP	-.035	.003	-.186*	-10.896	.000			
	UP	-.031	.005	-.137*	-6.247	.000			
	P	-.059	.015	-.203*	-4.050	.000			
	PGR	-.027	.009	-.099*	-3.108	.002			
	II	-.047	.009	-.159*	-5.178	.000			
	LS	-.011	.014	-.042	-.819	.413			
	SWC	-.038	.006	-.148*	-6.646	.000			
	U	-.036	.004	-.170*	-8.659	.000			

* Significant Predictors

Dependent Variable: Psychological Well-being

Independent Variables: ROL = Role Overload; RA = Role Ambiguity; RC = Role Conflict; UGPP = Unreasonable Group & Political Pressure; RP = Responsibility for Persons; UP = Under Participation; P = Powerlessness; PGR = Peer Group Relations; II = Intrinsic Improvishment; LS = Low Status; SWC = Strenuous Working Conditions; U = Unprofitability

## Discussion

The purpose of the study was to explore the relationship between perceived occupational stress and psychological well-being among secondary school heads in Khyber Pakhtunkhwa. A quantitative, descriptive and correlative research design was used to find out the relationship between perceived occupational stress and psychological well-being. A number of research studies have been conducted to examine the relationship between perceived occupational stress and psychological well-being of the employees in workplace [51–55, 61–64]. Similarly, the current study was carried out to investigate the relationship between the perceived occupational stress and psychological well-being among secondary school heads in Khyber Pakhtunkhwa. Research has explored that occupational stress has an adverse effect on mental health and quality of the organizational productivity [63]. Occupational stressors have pessimistic effects on the physical as well as psychological well-being and domestic life which make an individual to deviate from normal functioning. Unnecessary stress can cause some negative consequences i.e., sudden cardiac death, tuberculosis and diabetes, mental diseases like depression, despondency and anxiety and behavioural consequences such as unsatisfactory academic and work performance [65].

The article "Relationship between perceived occupational stress and psychological well-being among secondary school heads in Khyber Pakhtunkhwa, Pakistan" was retracted in 2025. Reasons: duplicated data; duplicated text; overlap with earlier publications; unreliable data.

The Pearson’s correlation analysis revealed that there is strong negative correlation between perceived occupational stress and psychological well-being. Additionally, the results revealed that there is moderate negative correlation between all the dimensions of perceived occupational stress and psychological well-being i.e. role overload, role ambiguity, role conflict, unreasonable group & political pressure, responsibility for persons, under participation, powerlessness, peer group relation, intrinsic improvishment, low status, strenuous working conditions, and unprofitability. The multiple linear regression analysis showed that 90% of the variance in psychological well-being is significantly represented by the independent variables. Furthermore, it was found that except low status low status, all the dimensions of perceived occupational stress have significant negative impact on psychological well-being. It plainly revealed that occupational stress has adverse effects on the psychological well-being of secondary school heads. The findings of the study are consistent with many research studies who also investigated the same results. Bell, Rajendran, and Theiler [66] noted that perceived occupational stress was strongly and negatively correlated with work life balance thus having a negative relationship to employees’ well-being but had a weaker positive relationship to the employees’ ill-being. Akintayo [67] concluded that occupational stress has a tendency to have a harmful effect on all areas of life, including the physical, psychosocial, social, intellectual and behavioral, which in turn affect the employees’ psychological well-being. There is a substantial impact of occupational stress on employees’ psychological well-being. Yunus and Bin Mahajar [52] found that there is a significant correlation between role ambiguity and psychological well-being. Likewise, Poormahmood, Moayedi, and Alizadeh [55] found a significant negative correlation between psychological well-being and occupational stress. Malek, Meanrns, and Flin [68] found that sources of occupational stress have significant negative correlations with job satisfaction and psychological well‐being. Kurnia [69] concluded that influence over decision, role clarity, autonomy and control, and peer support are the factors of stress at work which significantly impact employee’s psychological well-being. On the other hand, Ikonne [70] found that role ambiguity, role conflict, and work environment have a positive significant relationship on psychological well-being of the employees.

The article "Relationship between perceived occupational stress and psychological well-being among secondary school heads in Khyber Pakhtunkhwa, Pakistan" was retracted in 2025. Reasons: duplicated data; duplicated text; overlap with earlier publications; unreliable data.

## Conclusions

Conclusively, occupational stress is highly associated with psychological well-being having inverse relationship. The findings revealed that there is strong negative correlation between perceived occupational stress and psychological well-being among secondary school heads. Furthermore, there is moderate negative correlation between all the sub-scales of perceived occupational stress and psychological well-being. Except low status, each subscale of occupational stress has an adverse and negative effect on psychological well-being of secondary school heads. It means that psychological well-being is negatively affected by the occupational stress which leads to various negative consequences and affects the organizational achievements and productivity. Based on findings and conclusions, it was recommended that Elementary & Secondary Education Department should have a collaboration with policymakers to formulate a comprehensive strategy for stress reduction management for secondary school heads so that they may develop good psychological well-being and perform their duties effectively. Furthermore, trainings, seminars and workshops on psychological well-being and stress reduction management should be arranged for secondary school heads. Secondary school heads may be provided basic facilities and for this purpose, special budget should be reserved to improve the working conditions. They should be taken into confidence while formulating educational policies. They should be granted handsome compensation and other incentives. Political inference in school should be banned. In order to lessen the workload, a post of vice heads may also be created at secondary level.

## Supporting information

S1 Appendix Occupational stress index (OSI). (PDF)

S2 Appendix Raff’s psychological wellbeing scale (RPWS). (PDF)

S3 Appendix Permission letter from director of elementary & secondary education khyber pakhtunkhwa, pakistan for collecting data from government boys and girls schools. (DOCX)

S1 Data Set Data set regarding occupational stress and psychological wellbeing of secondary school heads. (XLSX)
